The article "Exploration of the Effect of Competence-Oriented Simulated Teaching Training on Comprehensive Competitiveness of Nursing Staff" was retracted in 2023. Reasons: signs of a paper mill; suspected computer-generated content; unreliable results or conclusions; lack of ethics approval or compliance.

# Exploration of the Effect of Competence-Oriented Simulated Teaching Training on Comprehensive Competitiveness of Nursing Staff

**DOI:** 10.1155/2022/9505764

**Published:** 2022-08-24

**Authors:** Ying Wang, Huifang Xu

**Affiliations:** Oncology Department, Zhejiang Hospital, Hangzhou 310030, China

## Abstract

In order to explore the effect of competence-oriented simulated teaching training on vocational theory, practice ability, learning effect, and postcompetence of nursing staff, a total of 107 inservice nursing staff in our hospital from January 2021 to September 2021 are selected and analyzed. They are divided into traditional group and simulated teaching group and received traditional explanation and demonstration training and ability oriented simulated teaching training, respectively. The experimental results show that the scores of vocational theory, practical operation ability, learning effect, and Competency Inventory for Registered Nurse (CIRN) of the simulated teaching group are significantly higher than those of traditional group. It is clearly evident that the competence-oriented simulation teaching method is beneficial to improve the professional theoretical level and practical ability of nursing staff. Also, the training method can improve the comprehensive learning ability and job competence.

## 1. Introduction

Nursing staff play an important role in clinical work. Strengthening the training of nursing staff can improve the quality of nursing work, so as to serve patients with high service quality [1, 2]. Conventional nursing training has a certain effect on improving theoretical knowledge and operational ability, but the quality of training is uneven [3]. Studies have shown that simulation teaching is more conducive to improve the quality of nursing. Through simulation teaching, nurses can simulate real clinical cases. Moreover, they can conduct indepth discussion and analysis on the problems existing in nursing, nursing methods, nurse patient relationship, etc. Therefore, nurses can further operate and cope with the actual situation on the basis of mastering theoretical knowledge so as to improve the overall working ability [4, 5]. Simulation teaching method can integrate the content that needs to be learned into complex situations so that nurses can use theoretical knowledge to solve problems. This will not only help nurses deepen their understanding of theoretical knowledge but also improve their practical ability so as to be better applied to clinical nursing work. Postcompetency can promote nurses to improve their theoretical and practical abilities, improve the quality and effect of nursing work, and promote nurses to achieve better results in their posts [6]. Therefore, it is necessary to take competence-oriented training combined with simulation teaching to further improve the comprehensive ability of nursing staff and enhance their postcompetence. However, there is still a lack of experimental data to support the clinical application effect of this teaching method [7]. Based on this, this study discusses and analyzes the influence of competence-oriented simulation teaching method on nursing staff's vocational theory, practical ability, and effect so as to provide reference for nursing staff training methods. The following reports are available.

The rest of this paper is organized as follows: Section 2 demonstrates the related work. Then, the research methods and observation indicators are presented in Section 3.  Section 4 presents the comparative results and analysis.  Section 5 concludes the paper.

## 2. Related Work

Through regular training, nurses can better carry out nursing work in clinical work [8]. For the daily training of nursing staff, teachers usually carry out indoctrination teaching for nursing staff according to the outline content, and the effect is poor [9]. Because it is difficult to integrate theory and practice, many nurses still have some difficulties in their work after returning to their posts after training [10, 11]. Different from the traditional training methods, the ability-oriented simulation teaching method can guide nurses to think about why and how to do it. It can help nurses apply theoretical knowledge to practice, help nurses get familiar with different working scenes, and help to improve theoretical knowledge and clinical nursing practice ability. In this way, nurses can be better qualified for their work [12].

Chen [13] suggested that the simulation teaching method can enhance the emergency handling ability of nursing staff and improve their practical ability, which is similar to the results of this study. In this study, the professional theory and practical operation scores of nursing staff in the simulated teaching group are improved more obviously after training, suggesting that the simulated teaching can improve the personal professional ability and training results of nursing staff. The reason may be that nurses deal with doctor-patient relationship and medical care relationship and participate in patients' rehabilitation activities through simulated teaching and exposure to simulated scenes. Communicating with doctors and patients in simulated scenarios can improve the communication ability of nursing staff and also contribute to the improvement of their humanistic qualities. Through simulation teaching, nursing staff's lateral thinking ability is greatly improved. It demonstrates that the training is helpful for them to correctly deal with emergencies and better combine their theoretical knowledge and practical ability [14].

The competence-oriented simulation teaching method can greatly improve the participation of nursing staff, stimulate their interest in learning, and improve their independent learning ability, thus contributing to the learning of theoretical knowledge. The adoption of simulation teaching and the introduction of real cases in the past can help the processing personnel improve their ability to deal with emergencies and improve their teamwork and communication skills [15]. The above results further suggested that the research team also believes that scenario simulation teaching can improve the nursing staff's various abilities and thus improve their comprehensive ability. In addition, the way of simulation to the simulation teaching faculty of higher overall satisfaction evaluation showed that the simulation of competence-oriented training way more recognition, analyzed its reason for training effect is remarkable, the quality of training content was higher, and finally realized the ability of the nursing staff, so nursing staff satisfaction was higher for the training.

Leung and Wang [16] showed that, through job competency training, nursing staff can better adapt to the work content and working environment and further improve the ability of nursing staff to be competent for work. The results of this study showed that compared with the traditional group, the postcompetency score of nursing staff in the simulated teaching group improved more obviously. It is analyzed that the mechanism may be competence-oriented training, which can evaluate nursing staff's various abilities and provide targeted training for their weak abilities. Nursing staff can also have a clearer understanding of their own abilities through competency scoring, which helped them better improve themselves and further strengthen their postcompetency, which was of great significance for them to carry out their work after returning to their posts [17, 18].

## 3. Data and Methods

### 3.1. General Information

A total of 107 in-service nursing staff in our hospital from January 2021 to September 2021 are selected as the training object, and 107 nursing staff are divided into traditional group and simulation group. The random number table method is used for grouping, including 53 people in the traditional group and 54 people in the simulation group. Among them, the traditional group is 19–25 years old with an average of 22.56 ± 2.33 years old. There are 2 males and 51 females, 27 with college degree and 26 with bachelor degree or above. The simulated teaching group is 19–25 years old, with an average age of 23.12 ± 1.47 years old. There are 4 males and 50 females, 33 with college degree and 21 with bachelor degree or above. There is no statistical difference between the two groups in age, gender, education level, and other general information (*P* > 0.05), indicating comparability. Inclusion criteria are as follows: (1) nursing staff internship time ≥6 months; (2) training times ≥5 times; (3) age ≥18; (4) those who know the contents of this study. Exclusion criteria are as follows: (1) leave ≥3 times during training; (2) nursing staff absent from duty due to sick leave; (3) nursing staff who go out for further study; (4) nursing staff who are unable to participate in the whole study due to work reasons.

### 3.2. Methods

Conventional training and teaching methods are applied to the traditional nursing staff. Teachers will explain conventional theoretical knowledge and demonstrate operation skills according to the training outline, and nursing staff will carry out theoretical learning and skill operation training according to the teacher's arrangement. After the training of nursing staff, it is necessary to participate in the unified organization assessment.

Based on routine training and teaching, the ability-oriented simulation teaching method was used to train the nursing staff in the simulation teaching group. Specific steps are as follows: (1) establish the training assessment group. The ability-oriented training model, training, and evaluation team should determine the postcompetitiveness of nursing staff according to the training objectives. Post competitiveness includes practical ability, critical thinking and scientific research ability, interpersonal skills, and ability indicators, such as professional development ability. The competency of each indicator is defined. Before the training, the assessment team can evaluate the competency of nursing staff, explain the evaluation results, and give guidance suggestions. Based on the competency assessment results, nursing staff will focus on training projects with weak capacity to ensure that the training content meets their own needs. At the end of the training, the assessment team should re-evaluate the competency of the nursing staff so that they can continue to improve themselves. (2) Under the guidance of teachers, the nursing staff will discuss and formulate specific scenario cases, collect clinical patients' complaints, general information, postoperative nursing and health education, and analyze the collected information and prepare scenario simulation cases. (3) According to the prepared situational simulation cases, the simulated teaching scenarios are arranged, including simulated wards, required equipment, and equipment. (4) Scenario simulation is conducted by grouping, with 9 people as one group and divided into 6 groups. The team members played roles according to the nurses, doctors, patients, and family members in the simulated cases, so that the nurses could enhance their ability to deal with the nurse-patient relationship and the relationship between doctors and nurses in the simulated teaching, and improve interpersonal communication and teamwork ability. Nursing staff should also take corresponding rehabilitation nursing for patients according to the situation of simulated cases, develop nursing plans, and implement according to the nursing plan, while making timely adjustments according to the actual situation of patients and feedback so as to promote the rehabilitation of patients. (5) After the simulation teaching, the teacher can analyze the problems existing in the simulation process of each group, guide the nursing staff to exchange their experience and learning experience, deepen their understanding of relevant theoretical knowledge and nursing measures, and strengthen their practical operation ability. The training cycle of the simulated teaching group is 8 weeks, once a week. Assessment is conducted at three time points before training, four weeks, and eight weeks during training, which are recorded as T1∼T3.

### 3.3. Observation Indicators and Evaluation Criteria

Observation indicators and evaluation criteria are as follows: (1) at the three observation points, closed-book examination and simulated practical operation are, respectively, adopted to evaluate the occupational theory and practical operation scores of the two groups of nursing staff, and the numerical differences are compared, with full marks of 100. (2) At three observation time points, questionnaire is used to evaluate the differences in learning effect, training satisfaction, and job competency scores of the two groups of nursing staff. The evaluation criteria of learning effect are as follows: independent learning ability, learning interest, comprehensive ability to deal with emergencies, teamwork ability, and communication ability, with a total score of 20 points for each item and a full score of 100 points. Nursing training satisfaction is evaluated by a satisfaction questionnaire made by our hospital. The scale included four options: very satisfied, satisfied, general, and dissatisfied. Cronbach's of the scale is 0.87, and the evaluation of satisfaction can be defined as: satisfaction = (number of very satisfied cases + number of satisfied cases)/total number of cases × 100%. The self-evaluated “Competency Inventory for Registered Nurse” (CIRN) is utilized, which included 7 dimensions and 58 items in total. Likert level 5 is used to score, with a total score of 0–232.

### 3.4. Statistical Treatment

SPSS 24.0 software is used to process the data in the study. The counting data are represented by *χ*^2^ test, the measurement data are represented by *t* test, and the mean ± standard deviation ($\bar{x}$ ± *s*) and the multiple groups of data are represented by *F* test. Mauchly test is employed to compare the results at different time points within the group. *P* > 0.05 indicated that the covariance matrix is full of football symmetry, and *P* < 0.05 indicated that the difference is statistically significant.

## 4. Results and Analysis

### 4.1. Vocational Theory Scores at Different Time Points

The occupational theory scores of the two groups showed an upward trend, the scores of T2 and T3 in the simulated teaching group are higher than those in the traditional group, and the data difference is statistically significant, as shown in Table 1 and Figure 1. The symbol “#” represents the comparison with the traditional group, *P* < 0.05.

### 4.2. Practical Operation Results at Different Time Points

The performance of the two groups showed an increasing trend, the performance of T2 and T3 in the simulation group is higher than that in the traditional group, and the data difference is statistically significant (*P* < 0.05), as shown in Table 2 and Figure 2.

### 4.3. Score of Learning Effect at Different Time Points

The learning effect scores of the two groups shows an increasing trend. The scores of T2 and T3 in the simulated teaching group are higher than those in the traditional group, and the data difference is statistically significant (*P* < 0.05), as shown in Table 3 and Figure 3.

### 4.4. Comparison of Training Satisfaction Difference

The training satisfaction of the simulated teaching group and the traditional group is 96.30% and 58.49%, respectively. The training satisfaction of the traditional group is lower than that of the simulated teaching group, and the data difference is statistically significant (*P* < 0.05), as shown in Table 4. It demonstrates that the competence-oriented simulated teaching training model can not only deepen their understanding and memory of theoretical knowledge but also improve their practical operation ability.

### 4.5. Changes of Postcompetency Scores at Different Time Points

The job competency scores of the two groups showed an upward trend, the scores of T2 and T3 in the simulated teaching group are higher than those in the traditional group, and the data difference is statistically significant (*P* < 0.05), as shown in Table 5 and Figure 4. After training, most nurses in the simulated teaching group showed significant improvement in autonomous learning ability and comprehensive ability to deal with emergencies and teamwork ability. Analysis of the reason may be that the previous routine training is boring, nursing staff learning interest and enthusiasm are not high, so the learning effect is poor.

## 5. Conclusions and the Future Work

In this study, a total of 107 in-service nursing staff are selected and analyzed to explore the effect of competence-oriented simulated teaching training on vocational theory, practice ability, learning effect, and postcompetence. The experimental results show that the scores of vocational theory, practical operation ability, learning effect, and Competency Inventory for Registered Nurse (CIRN) of the simulated teaching group are significantly higher than those of traditional group. It is clearly evident that the competence-oriented simulation teaching method is beneficial to improve the professional theoretical level and practical ability of nursing staff. Also, the training method can improve the comprehensive learning ability and job competence. The competence-oriented simulation teaching method for nursing staff training can obtain the good teaching effect and achieve a significant boost to enhance the quality of nursing work. However, there are still shortcomings in this study. Although the simulated teaching method can simulate the working scenes of nursing staff and emergencies more realistically, there is still a certain gap with the real clinical scene. In addition, the sample size is small, and further exploration is required to provide reference for nursing staff training.

## Figures and Tables

**Figure 1:** Changes of vocational theory scores at different time points.

**Figure 2:** Variation of practical operation results at different time points.

**Figure 3:** Changes in learning effect scores at different time points.

**Figure 4:** Changes of postcompetency score at different time points.

**Table 1:** Occupational theory scores at different time points ($\bar{x}$ ± *s*).

Group	Time point	Career theory results
Simulation teaching group (*n* = 54)	T1	53.52 ± 3.54
	T2	80.52 ± 4.34
	T3	91.23 ± 5.63
Traditional group (*n* = 53)	T1	53.49 ± 3.23
	T2	67.52 ± 4.43
	T3	82.26 ± 5.35
*F *_time point_		433.515
*P *_time point_		<0.001
*F*_point*∗*group_		514.322
*P*_point*∗*group_		<0.001

**Table 2:** Practical operation results at different time points ($\bar{x}$ ± *s*).

Group	Time point	Practice performance
Simulation teaching group (*n* = 54)	T1	54.56 ± 2.23
	T2	81.55 ± 3.32
	T3	92.24 ± 4.83
Traditional group (*n* = 53)	T1	54.53 ± 2.19
	T2	72.32 ± 3.23
	T3	87.43 ± 3.44
*F *_time point_		423.511
*P *_time point_		<0.001
*F*_point*∗*group_		543.353
*P*_point*∗*group_		<0.001

**Table 3:** Score of learning effect at different time points ($\bar{x}$ ± *s*).

Group	Time point	Learning effect score
Simulation teaching group (*n* = 54)	T1	48.23 ± 3.11
	T2	75.63 ± 4.12
	T3	89.53 ± 4.44
Traditional group (*n* = 53)	T1	48.19 ± 3.09
	T2	64.43 ± 4.02
	T3	78.35 ± 4.32
*F *_time point_		413.453
*P *_time point_		<0.001
*F*_point*∗*group_		512.544
*P*_point*∗*group_		<0.001

**Table 4:** Comparison of training satisfaction differences (*n*, %).

Divide into groups	Example number	Very satisfied	Satisfied	Just like	Discontent	Degree of satisfaction
Traditional group	53	13	18	21	1	31
Simulation teaching group	54	49	3	2	0	52
*x * ^2^	—	—	—	—	—	11.247
*P*	—	—	—	—	—	0.016

**Table 5:** Changes of postcompetency scores at different time points ($\bar{x}$ ± *s*).

Group	Time point	Job competency score
Simulation teaching group (*n* = 54)	T1	138.23 ± 23.55
	T2	165.63 ± 30.34
	T3	199.53 ± 42.44
Traditional group (*n* = 53)	T1	138.17 ± 23.47
	T2	154.43 ± 27.24
	T3	178.83 ± 37.34
*F *_time point_		465.456
*P *_time point_		<0.001
*F*_point*∗*group_		512.544
*P*_point*∗*group_		<0.001

## Data Availability

The simulation experiment data used to support the findings of this study are available from the corresponding author upon request.

## References

[1] Wang L., Guo J. Y., Sun H. (2021). Construction and application of nurses’training system in emergency department based on learning organization Theory. *Nursing Management*.

[2] Cer A., Vnbn B., Eo A. (2021). The effectiveness of extended-duration supervision training for nurses and allied health professionals: a realist evaluation. *Nurse Education Today*.

[3] Doughty L., Sinnema C., Mckillop A., Dixon R. (2021). The impact of postgraduate education in transition to practice programs on new graduate nurses’ knowledge and skills: a pre-post survey design. *Nurse Education Today*.

[4] Naggar M. A. E., Almaeen A. H. (2020). Student’s perception towards medical-simulation training as a method for clinical teaching. *JPMA. The Journal of the Pakistan Medical Association*.

[5] Daoud I. M. M., Suliman A. G., Abdelrahim A., Mohammed M. M. E., Mohammed N. E. (2020). Simulation based learning versus clinical rounds in hospitals as a method of teaching in obstetrics. *Australasian Medical Journal*.

[6] Jia X., Gong S. W., Liu J. Y. (2020). The application of stage goal teaching combined with situational simulation training in the teaching of CCU practice nurses. *Chinese journal of modern nursing*.

[7] Chen Q. Q., Mou S. Y., Zhang C. L. (2021). Practice of standardized training of nurses for clinical teachers based on teaching competence. *Chinese Journal of Medical Education*.

[8] Baker J. K. R., Flores B. E., Caughan S. Y. M. (2020). Outcomes educating nursing students using an evolving, Simulated Case Scenario. *Clinical Simulation in Nursing*.

[9] Zhang W. Q., Gao W. J. (2021). Application status and prospect of core competence scale for registered nurses in China. *Hainan Med*.

[10] Chen H., Feng H., Liao L. (2020). Evaluation of quality improvement intervention with nursing staff training in nursing homes: a systematic review. *Journal of Clinical Nursing*.

[11] D’Souza P., George A., Nair S., Noronha J., Renjith V. (2021). Effectiveness of an evidence-based practice training program for nurse educators: a cluster-randomized controlled trial. *Worldviews on Evidence-Based Nursing*.

[12] Gao Y., Sun H. M., Pei S. Q. (2020). Construction and practice of training program for blood purification specialized nurses based on job competency. *Chinese journal of modern nursing*.

[13] Chen J. (2022). Application analysis of nurse-patient cooperative situation simulation teaching in basic first-aid technical nursing. *Modern Digestive and Interventional Diagnosis and Treatment*.

[14] Huang D. H., He L. J., Shi Q. L. (2021). Management and practice of specialized nurses based on post competency. *Journal of Nursing Education*.

[15] Zo A., Emm B., Unger R. S. (2022). Enhancing the structural competency of nurses through standardized patient simulation. *Clinical Simulation in Nursing*.

[16] Leung M. F., Wang J. (2022). Cardinality-constrained portfolio selection based on collaborative neurodynamic optimization. *Neural Networks*.

[17] Chan T. E., Lockhart J. S., Thomas A., Kronk R., Schreiber J. B. (2020). An integrative review of nurse practitioner practice and its relationship to the core competencies. *Journal of Professional Nursing*.

[18] Yu Y., Rashidi M., Samali B., Yousefi A. M., Wang W. (2021). Multi-image-feature-based hierarchical concrete crack identification framework using optimized SVM multi-classifiers and D–S fusion algorithm for bridge structures. *Remote Sensing*.

